The article "Potential Impact of Multi-Walled Carbon Nanotubes Exposure to the Seedling Stage of Selected Plant Species" was retracted in 2015. Reasons: plagiarized text; duplicated text; overlap with other authors' work; overlap with earlier publications.

# Potential Impact of Multi-Walled Carbon Nanotubes Exposure to the Seedling Stage of Selected Plant Species

**DOI:** 10.3390/nano4020203

**Published:** 2014-03-31

**Authors:** Parvin Begum, Refi Ikhtiari, Bunshi Fugetsu

**Affiliations:** Laboratory of Environmental Medical Chemistry, Graduate School of Environmental Science, Hokkaido University, Sapporo 060-0810, Japan; E-Mails: refi@ees.hokudai.ac.jp (R.I.); hu@ees.hokudai.ac.jp (B.F.)

**Keywords:** phytotoxicity, multi-walled carbon nanotubes (MWNTs), seedling stage, cell death, electrolyte leakage

## Abstract

Phytotoxicity is a significant consideration in understanding the potential environmental impact of nanoparticles. Abundant experimental data have shown that multi-walled carbon nanotubes (MWNTs) are toxic to plants, but the potential impacts of exposure remain unclear. The objective of the present study was to evaluate possible phytotoxicity of MWNTs at 0, 20, 200, 1000, and 2000 mg/L with red spinach, lettuce, rice, cucumber, chili, lady’s finger, and soybean, based on root and shoot growth, cell death, and electrolyte leakage at the seedling stage. After 15 days of hydroponic culture, the root and shoot lengths of red spinach, lettuce, and cucumber were significantly reduced following exposure to 1000 mg/L and 2000 mg/L MWNTs. Similar toxic effects occurred regarding cell death and electrolyte leakage. Red spinach and lettuce were most sensitive to MWNTs, followed by rice and cucumber. Very little or no toxic effects were observed for chili, lady’s finger, and soybean.

## 1. Introduction

The production of engineered nanomaterials is a scientific breakthrough in material design and nanoscience has developed significantly during the last decade as it has transitioned from worktable top science to applied technology [1]. Multi-walled carbon nanotubes (MWNTs) are a type of nanomaterials that have attracted remarkable interest in terms of both fundamental research and technological development [2] due to their unique nanostructures and extraordinary properties (high electrical conductivity, large specific surface area, high aspect ratio and remarkable thermal stability) [3]. Hundreds of nanotechnology-based products are currently in the marketplace, with common applications in agriculture, food production, food packaging, and food protection [4]. Promising applications in a wide variety of areas (medicine, pharmaceuticals, manufacturing technologies, electronics and telecommunications) using nanomateials are being developed rapidly [5]. The forecasted huge increasing use of nanoparticles in industrial and household applications makes it likely that increasing human and environmental exposure to nanoparticles will occur [6]. Furthermore, at the end of their life cycle, most nanotechnology products are disposed in landfills or intentionally put into the soil to assist soil and groundwater remediation. Consequently, nanomateials may be released into the soil–water system [7]. Scientists agree that the spread of nano-scale products will be beneficial to science, medicine and technology, but their release into the environment might cause adverse health effects to humans, living organisms and sensitive ecosystems [8,9]. Governmental agencies, including the United States National Institute for Occupational Safety and Health and Japan's Ministry of Health, have recently raised the question of whether apparently harmless materials such as carbon-based nanotubes should be treated with the same caution afforded known carcinogens such as asbestos [10].

The article "Potential Impact of Multi-Walled Carbon Nanotubes Exposure to the Seedling Stage of Selected Plant Species" was retracted in 2015. Reasons: plagiarized text; duplicated text; overlap with other authors' work; overlap with earlier publications.

To address this issue, a number of investigators around the earth have taken initiative to reveal the phenomena of phyto-toxity of nanomaterials. Plants comprise a very vital living component of terrestrial ecosystems, provide a potential pathway for the transport of nanomaterials to the environment and serve as an important route for their bioaccumulation into food chain [11]. Phyto-toxicity evaluation holds the promise of controlled use of nanoparticles [11]. However, until now, studies of the interactions between nanomaterials and plants have been largely overlooked, and most of the publications are limited to explanations of phenomena observed. On one hand, previous research has shown that nanomaterials will influence plant growth and development. On the other, plant metabolic activities will affect transformation and fate of nanomaterials in the environment in addition to their transportation in food chain [12]. Nanomaterials have been shown to generate harmful reactive oxygen species (ROS) due to their large surface areas, thus increasing cellular oxidative stress and possibly attacking DNA, proteins, and membranes, resulting in cellular injury [5]. The novel and extraordinary physiochemical properties such as their size, shape, surface properties and their unique characteristics raise growing concerns regarding potentially adverse effects on biological and ecological systems [1]. We therefore emphasized the necessity to assess for future research on toxicological effect, with specific emphasis on plants, before introducing nanoproducts into the marketplace.

The threshold at which signs of toxicity become established differs widely among plant species, and the impact of nanoparticles on different plant species can vary greatly, depending on the plant growth stage and the method and duration of exposure, as well as on nanoparticle size, concentration, chemical composition, surface structure, solubility, shape, and aggregation [13]. The varying experimental conditions used in different studies make it difficult to strictly classify plants into tolerance groups. Some broad generalizations are possible, but there is a vital need to examine the possible toxicity of nanomaterials to diverse crop species.

The article "Potential Impact of Multi-Walled Carbon Nanotubes Exposure to the Seedling Stage of Selected Plant Species" was retracted in 2015. Reasons: plagiarized text; duplicated text; overlap with other authors' work; overlap with earlier publications.

In terms of phytotoxicity, several studies have focused on terrestrial plant species exposed to MWNTs [14,15], but no continual, full, or multigenerational life-cycle studies appear in the literature, demonstrating the need for wide-ranging study of interactions between carbon nanoparticles and terrestrial plants, as well as the ultimate fates of exposed plants. To address this need, we investigated the interaction between MWNTs and the vegetable/commercial crops, red spinach, lettuce, rice, cucumber, chili, lady’s finger, and soybean, focusing on root and shoot growth and cell death at the seedling stage [16]. The most sensitive plant species were then used in phytotoxicity studies in the presence of MWNTs. Our experiment demonstrated that red spinach, lettuce, rice, and cucumber experience much higher toxicity from MWNTs at the seedling stage, indicating the need for further research including a wide range of terrestrial plant species associated with carbon nanoparticles and this approaches to improve nano safety screening.

## 2. Results and Discussion

### 2.1. MWNTs Analysis

MWNTs were characterized based on the various techniques such as scanning electron microscope (SEM), transmission electron microscope (TEM), atomic force microscopy (AFM) and inductively coupled plasma mass spectrometer (ICP-MS, Seiko-SPQ-6500, Shimadzu, Tokyo, Japan) have been performed. Figure 1 shows the (a) SEM, (b) TEM micrographs of MWNTs before and after suspended in a modified Hoagland medium, and (c) AFM image of MWNTs before suspended in a modified Hoagland medium, represents the morphology of the water-wetted milled MWNTs that were used in this study. Details information about the metals content come from ICP-MS analysis, paying attention to the relative metal (Fe, Co, Ni, Mn and Cr) concentrations of MWNTs. Information on quantitative analysis of the metal impurities (ppm in weight) for MWNTs before and after suspended in a modified Hoagland medium, we obtained below the detection limit of Fe, Co, Ni, Mn and Cr, only in modified Hoagland medium, Fe = 174.53 and Mn = 455.75, because the hydroponic solution containing the Fe and Mn.

### 2.2. MWNTs Induced Morphological Changes in Plants

The physiology and morphology of red spinach, lettuce, rice, cucumber, chili, soybean, and lady’s finger were assessed following hydroponic culture with MWNTs. The effects of MWNTs exposure at 20, 200, 1000, and 2000 mg/L on shoot and root growth varied by plant species (Figure 2). MWNTs showed no toxic effects on chili, lady’s finger, or soybean (data not shown), but the root and shoot growths of lettuce, red spinach, cucumber, and rice were reduced compared to control. The MWNTs-treated plants displayed a gradual change in leaf color to light green/yellowish with increasing MWNTs dose (lettuce, rice, Figure 2); untreated plants (control) did not exhibit any change in color (lettuce, rice, Figure 2) compared to MWNTs-treated plants. Wilting of leaves of reduced size was evident by visual observation in MWNTs-treated red spinach, lettuce, and rice (Figure 2). The attachment of MWNTs to plant roots was characterized by visual observation (Figure 2).

The article "Potential Impact of Multi-Walled Carbon Nanotubes Exposure to the Seedling Stage of Selected Plant Species" was retracted in 2015. Reasons: plagiarized text; duplicated text; overlap with other authors' work; overlap with earlier publications.

**Figure 1:** (**a**) SEM (Bar: 500 nm); (**b**) TEM (Bar: 200 nm) micrographs of MWNTs before and after suspended in a modified Hoagland medium; and (**c**) AFM image of MWNTs before suspended in a modified Hoagland medium, depicts the morphology of MWNTs. Reproduced with permission from reference [17], Copyright 2012, Elsevier.

**Figure 2:** Morphological observations of red spinach, lettuce, rice, and cucumber exposed to MWNTs at 0, 20, 200, 1000, or 2000 mg/L for 15 days. Reproduced with permission from reference [16], Copyright 2012, Elsevier.

Rice is a monocot, and the other tested species are dicots; the seeds of red spinach, lettuce, and cucumber are smaller than those of soybean and lady’s finger. Red spinach and lettuce have the smallest seed sizes and displayed the greatest phytotoxicity among the seven species tested here. Seed size can be an important factor in how a seed responds to MWNTs. For example, small-seeded species have a large surface area to volume ratio, which is conducive to higher sensitivity to toxicants [18] than large-seeded species such as lady-finger and soybean. Size may therefore cause seeds to be more sensitive to nanoparticle exposure, but it does not dictate whether phytotoxicity will be experienced.

### 2.3. Effects of MWNTs on the Growth of Plants

The root and shoot growth of red spinach, lettuce, rice, and cucumber exposed to MWNTs at 2000 mg/L were significantly different from the control plants (Figure 3). The reductions in shoot fresh weight of red spinach, lettuce, rice, and cucumber plants at 2000 mg/L exposure were 88%, 63%, 46%, and 36%, respectively (Figure 3a,b). Interestingly, the shoot fresh weight of rice was reduced 56% at 20 mg/L and 46% at 2000 mg/L compared to control (Figure 3a). Red spinach, lettuce, and cucumber shoot heights at 2000 mg/L exposure decreased by 80%, 50%, and 66%, respectively (Figure 3c), and the shoot length of rice was reduced by 48% at 20 mg/L and by 35% at 200 mg/L compared to control (Figure 3c).

The article "Potential Impact of Multi-Walled Carbon Nanotubes Exposure to the Seedling Stage of Selected Plant Species" was retracted in 2015. Reasons: plagiarized text; duplicated text; overlap with other authors' work; overlap with earlier publications.

The root fresh weights of red spinach and lettuce at 2000 mg/L declined 81% and 79%, respectively (Figure 3d). The average root fresh weight of untreated rice was 0.0173 g, while the weights of treated rice at 20, 200, 1000, and 2000 mg/L MWNTs were 0.0063, 0.004, 0.0037, and 0.0036 g, respectively (Figure 3d). The average root fresh weight of control cucumber was 0.405 g, and the average root weight of treated cucumber decreased to 0.395, 0.36, 0.24, and 0.22 g following exposure to 20, 200, 1000, and 2000 mg/L MWNTs, respectively (Figure 3e). The reductions in the root lengths of red spinach and lettuce at 2000 mg/L exposure were 67% and 45%, respectively (Figure 3f). The average root length of untreated rice was 5.3 cm, and those of treated rice were 6, 4.7, 6.83, and 5.5 cm at 20, 200, 1000, and 2000 mg/L MWNTs, respectively. The reduction in shoot and root growth for rice was not in a concentration-dependent manner. The average root length of untreated cucumber was 10 cm, a length that decreased to 8, 8.7, 6.3, and 9.5 cm following exposure to 20, 200, 1000, and 2000 mg/L MWNTs, respectively (Figure 3f).

Growth (root, shoot length, and biomass) decrease is the most general symptom of MWNTs toxicity in the studied plants. Exposure to MWNTs at 1000 mg/L and 2000 mg/L resulted in significant decreases in red spinach and lettuce root and shoot growth compared to untreated plants. These observations are in agreement with those of Stampoulis *et al*. [19], who exposed zucchini to MWNTs at 1000 mg/L for two weeks. Our observation of a decrease in the number of leaves (data not shown) corresponds to inhibition of *Arabidopsis thaliana* growth [20]. The number of leaves has been used as a phytotoxicology endpoint for nanomaterials. Significantly fewer leaves (3 leaves) were present on red spinach exposed to 1000 mg/L and 2000 mg/L MWNTs (Figure 2) compared to control, corroborating the potential phytotoxicity of MWNTs. All control red spinach developed seven leaves each and retained red and healthy during the 15 days, whereas treated (1000 mg/L and 2000 mg/L) plants exhibited reduced leaf number and area and altered leaf shape, as the area was more suppressed than the length. Lin *et al.* [21] reported the positive effects of suspensions of MWNTs on seed germination and root growth of six different crop species (radish, rape, rye grass, lettuce, corn and cucumber). Lahiani *et al.* [22] found the positive effect of MWNTs on the seed germination and growth of seedlings of three important crops (barley, soybean and corn). In Zucchini plants, no negative effects were observed on seed germination and root elongation in the tested range of MWNTs; however, a decrease in the biomass of plants was observed during further growth in the presence of SWNTs [19].

The article "Potential Impact of Multi-Walled Carbon Nanotubes Exposure to the Seedling Stage of Selected Plant Species" was retracted in 2015. Reasons: plagiarized text; duplicated text; overlap with other authors' work; overlap with earlier publications.

**Figure 3:** Growth reduction of red spinach, lettuce, rice, and cucumber after 15 days of exposure to MWNTs. (**a**,**d**) Shoot and root weights, respectively, of red spinach, lettuce, and rice. (**b**,**e**) Shoot and root weights, respectively, of cucumber. (**c**,**f**) Shoot and root lengths, respectively, of red spinach, lettuce, rice, and cucumber. Error bars represent standard deviation of the mean (*n* = 3). The cucumber data are presented separately because the shoot and root fresh weights were larger than for the other tested plants. Reproduced with permission from reference [16], Copyright 2012, Elsevier.

### 2.4. MWNTs Induces Cell Death and Membrane Damage in Plants

We used the Evans blue staining method to detect cell death in 15-day-old fresh roots grown hydroponically with 0–2000 mg/L MWNTs. The absorbance measurement of the Evans blue extracted from roots showed a concentration-dependent manner (Figure 4a). With the concentration of MWNTs increasing to 1000 and 2000 mg/L in the case of red spinach, the amount of Evans blue uptake in root cells increased by about 7.9 and 12.0 fold, respectively, compared to that of control roots. Higher (1000 and 2000 mg/L) MWNTs concentrations also caused severe stress on plant growth and biomass (Figure 2 and Figure 3). We also used electrolyte leakage, an indicator of membrane damage, to show the extent of cell death. At 20 mg/L and 200 mg/L MWNTs, the leaves displayed little increase in electrolyte leakage after 15 days of exposure, while 1000 mg/L and 2000 mg/L exposure led to a drastic increase in electrolyte leakage (Figure 4b), reflecting dose-dependent electrolyte leakage. ROS accumulation reportedly causes cell death that can be demonstrated by electrolyte leakage from cells and rapid rise of Evans blue uptake [17,23]. Hence, the present findings suggest that intracellular ROS might have a crucial role in MWNTs-mediated induction of cell death.

**Figure 4:** Dose dependency of (**a**) cell death and (**b**) membrane integrity caused by 15-day exposure to MWNTs at 0, 20, 200, 1000, or 2000 mg/L in red spinach, lettuce, rice, and cucumber roots. Error bars represent standard deviation of the mean (*n* = 3). Reproduced with permission from reference [16], Copyright 2012, Elsevier.

A number of investigations have indicated that ROS (reactive oxygen species) generation and oxidative stress are mechanisms of MWNTs-induced plant toxicity. MWNTs-induced stress at 1000 mg/L and 2000 mg/L caused cell death and membrane damage in red spinach, lettuce, rice, and cucumber after 15 days of exposure, suggesting that MWNTs may induce ROS formation, promoting cell death and electrolyte leakage in the root and leaf, respectively. MWNTs aggregation was noted on the root surfaces, contributing at least a portion of the toxic effects of MWNTs [24]. Root hairs and root tips produce great amounts of mucilage, a highly hydrated polysaccharides covering on the root surface [25], which are the key species accountable for absorbing the nanoparticles onto root surface. Once CNTs accumulated on the cell walls will be having a plenty of chances to interact with the proteins and/or polysaccharides [24]. Many researchers believe that the detected toxicity of nanoparticles in plants is based on plant-nanoparticles physical interactions. The presence of nanoparticles on the root surface could modify the surface chemistry of the root such that it effects on how the roots interact with its environment [14].

The article "Potential Impact of Multi-Walled Carbon Nanotubes Exposure to the Seedling Stage of Selected Plant Species" was retracted in 2015. Reasons: plagiarized text; duplicated text; overlap with other authors' work; overlap with earlier publications.

### 2.5. MWNTs Induces ROS Generation in Red Spinach

Red spinach seedlings were somewhat more sensitive to MWNTs among the seven species tested here. To determine whether MWNTs can facilitate generation of excess ROS in MWNTs-treated red spinach, we used ROS-sensitive dyes (NBT, DAB and DCFH-DA) to evaluate the ROS accumulation induced by MWNTs in 15-day-old fresh red spinach leaves for further study. Compared to controls (Figure 5a,c), infiltration of MWNTs-treated leaves with DAB and NBT resulted in deep reddish-brown polymerization (Figure 5b) and blue formazon (Figure 5d) respectively. This indicated the accumulation of super oxide, and H_2_O_2_ respectively, in which the respective production rates were larger than the detoxification rates.

**Figure 5:** Detection of ROS in red spinach leaves. 15 day-old fresh leaves treated with or without MWNTs (0 and 1000 mg/L) were used for all measurements. (**a**,**b**) Staining using the 3–3'-diaminobenzidine (DAB) (Image obtained with a magnification of 4×). The brown staining indicates the formation of a brown polymerization product when H_2_O_2_ reacts with DAB, and viewed with light microscopy. (**c**,**d**) Staining using the NBT (Image obtained with a magnification of 4×). The blue staining indicates the formation of a blue formazon product when superoxide reacts with NBT, and viewed with light microscopy. (**e**,**f**) Staining with DCFH-DA (Image obtained with a magnification of 4×). The green signal indicates the presence of hydroperoxides inside the cells. Leaves were observed with fluorescence microscopy.

The article "Potential Impact of Multi-Walled Carbon Nanotubes Exposure to the Seedling Stage of Selected Plant Species" was retracted in 2015. Reasons: plagiarized text; duplicated text; overlap with other authors' work; overlap with earlier publications.

Infiltration of leaves with DCFH-DA allowed the detection of hydroperoxides. In untreated leaves there were few cells with fluorescence spots (Figure 5e); fluorescence spots were start increased with increasing MWNTs level (1000 mg/L) (Figure 5f), meaning that more cells were stressed and dead. This confirmed the results of NBT and DAB staining, that vascular bundles were experiencing oxidative stress. These results show a contribution of ROS in MWNTs-induced cell death and correspond to previous findings regarding MWNTs-potentiated ROS production in rice cell suspension [23]. Our results show that MWNTs elicit ROS production that appears to be required for phytotoxicity and precedes cell death via an apoptotic pathway or by necrosis.

ROS generation assessed by DCFH-DA, DAB, and NBT confirmed the direct presence of ROS generated inside the leaf in red spinach grown with MWNTs. Ascorbic acid prevented the increase in ROS generation in red spinach leaf [26], also confirmed that MWNTs induces ROS. The MWNTs-treated red spinach plants exhibited toxic symptoms with severely decreased plant growth after 15 days exposure, whereas plants treated with MWNTs and AsA exhibited normal growth, similar to the Hoagland medium only. Induction of cell death, membrane damage through generation of ROS in red spinach could be supported by the internalization of the MWNTs into the cells [26]. Accumulation of MWNTs on plant cell tissues might alter the plant physiological processes, including disruption of membrane integrity. ROS generation and rapid cell death are all characteristics of hypersensitive response (HR) [27]. Plants continuously produce ROS as byproducts of various metabolic pathways, e.g., mitochondria, chloroplasts, and peroxisomes are the main organellar producers of ROS [28]. It reported previous studies that MWNTs was capable of generating ROS to plant cell [23,24,29]. However, contact between cells and nanoparticles can also induce release of ROS. Appropriate proportions of molecular oxygen and various antioxidants required for cell survival. Reactive products of oxygen are amongst the most potent threats faced by cells. Generally, there exists equilibrium between pro-oxidant species and antioxidant defense mechanisms. ROS can induce cell death, when the cell’s antioxidant defenses are overwhelmed. ROS can cause damage to all of the major classes of biological macromolecules, including carbohydrates, nucleic acids, proteins, and lipids [30,31]. Due to their small size and high surface reactivity, the nanopaticles can cross most of the biological barriers and interact with intracellular structures, contribute to potential cellular and genetic toxicity by the induction of oxidative stress [32,33].

The article "Potential Impact of Multi-Walled Carbon Nanotubes Exposure to the Seedling Stage of Selected Plant Species" was retracted in 2015. Reasons: plagiarized text; duplicated text; overlap with other authors' work; overlap with earlier publications.

### 2.6. Morphological Observation of Red Spinach Roots and Leaves Using SEM

The changes in surface morphology of the red spinach leaf after MWNTs (1000 mg/L) exposure were studied through SEM (Figure 6). The SEM micrograph for untreated leaf shows a normal smooth surface, most stomata identified as open (Figure 6a,c). After MWNTs treatment for 15 days, the smoothness of the surface disappeared and surface displayed a remarkable range of changes in the morphology such as swelling and rupture (Figure 6b,d). Most stomata of the MWNTs-treated red spinach leaves were identified as closed by SEM analysis (Figure 6b). Stomata closure prevents water loss [34], leading to a reduced CO_2_ concentration inside the leaf. Pathogen-infected guard cells may close their stomata via a pathway involving H_2_O_2_ production [35], thus interfering with the constant attack of pathogens through the stomatal pores. Lee *et al.* [35] investigated how guard cells respond to elicitors that can be created from cell walls of plants or pathogens through pathogen infection. They tested the effects of elicitors (oligogalacturonic acid (OGA), a degradation product of the plant cell wall, and chitosan (β-1,4-linked glucosamine), a component of the fungal cell wall) on stomatal movements in tomato plant species. They found that elicitors induce the production of ROS in guard cells and to reduce stomatal aperture either by inhibiting stomatal opening or by inducing stomatal closing. Stomatal opening provides access to inner leaf tissues for many plant pathogens, so contraction stomatal openings may be advantageous for plant defense. Plants normally activate a variety of defense mechanisms against pathogen infection, often leading to production of ROS, such as superoxide and H_2_O_2_, which can in turn facilitate a HR [36]. McAinsh *et al.* [37] observed that exogenously added H_2_O_2_ and superoxide prevent stomatal opening and stimulate stomatal closing.

**Figure 6:** SEM observation of the red spinach leaf grown *in vivo* for 15 days in a medium containing Hoagland media only (control) and supplemented with 1000 mg/L MWNTs (treated). Image showing the morphology of control leaf (**a**,**c**) epidermis and MWNTs treated leaf (**b**,**d**) epidermis showing swelling epidermis. SEM observation of red spinach roots grown *in vivo* for 15 days in a medium containing Hoagland media only (control, **e**) and supplemented with 1000 mg L^−1^ MWNTs (treated, **f**) showing deformed root cap and elongation zone and deformed epidermis. Bar: **a** and **b**, 60 µm; **c** and **d**, 15 µm; **e**, 150 µm; **f**, 429 µm.

The root surfaces of the control plants, observed by SEM, were properly developed (Figure 6e). With MWNTs (1000 mg/L), the outer cell layers forming the epidermis underwent the greatest changes (Figure 6f). Many root cells exhibited damaged cell walls and root cap, cracks, loss of tissue, and the detachment of the outer cell layers (Figure 6f).

The article "Potential Impact of Multi-Walled Carbon Nanotubes Exposure to the Seedling Stage of Selected Plant Species" was retracted in 2015. Reasons: plagiarized text; duplicated text; overlap with other authors' work; overlap with earlier publications.

Despite different nanomaterial lengths and diameters [19], as well as the use of a variety of experimental techniques such as sonication [24] and functionalization [14], MWNTs have been consistently shown to aggregate and exert adverse effects in plants and plant cells. Functionalization of nanoparticles or the coating of the surface by natural compounds is clearly an important process in the environment which has, however, been studied only marginally so far. Functionalized nanoparticles changed their behavior significantly. Exposure scenarios with functionalized engineered nanoparticles that are primarily used in technical applications rather than pristine engineered nanoparticles should be investigated and could be applicable for evaluating impacts on the environment [38]. In a study by Says *et al.* [39] carbon nanoparticle functionalization led to a remarkable decline in toxic effects. Lin *et al.* [40] observed that both the pristine and HCL treated MWNTs were toxic to Arabidopsis T87 suspension cells. The studies by Miralles *et al.* [41] in wheat and alfalfa established that uptake of Fe_3_O_4_-functionalized MWNTs in the epidermis of wheat root tip is possible, not in alfalfa. They found that two crop species, alfalfa and wheat, were not damaged by MWNTs. Our experimental data indicate that MWNTs are toxic to red spinach, lettuce, rice, and cucumber, but not to chili, lady’s finger, and soybean. Physiological endpoint such as germination and morphological endpoints such as plant height, biomass and visual appearance of plants were used to accomplish this research. These are useful for obtaining evidence of possible toxicity symptoms. Chili, lady’s finger, and soybean did not respond to the exposure at 2000 mg/L. Some other studies also support the positive effects of suspensions of MWNTs [42]. MWNTs have been shown to penetrate thick seed coats, stimulate germination, and activate enhanced growth in tomato plants. The nanoparticles actually effect total gene expression. For example, the water channel gene is up-regulated in tomato seedlings with exposure to MWNTs. Plants of different species respond with their very own behaviors to the nanoparticles. Difference in structures of the xylem would be the key physiological reason responsible for this fact [23]. Based on several studies of nanoparticles, the following are the principal factors that influenced toxicity in agricultural food crops: nanoparticle size and specific surface area of nanoparticle, nanoparticles stability, plant species, growth media, dilution agent, *etc.* [13,43]. The size of seeds of the plant and root anatomy could render more sensitivity to nanoparticles exposure. Due to differences in root anatomy, xylem structures determine the speed of water transport, and different xylem structures may demonstrate different uptake kinetics of nanoparticle [12,14]. Xylem structure (ring-porous, semi-ring-porous, diffuse-porous) is a critical character in the adaptation of plant to variation in the environment. Xylem is sensitive to water stress, and responses to water stress in ring-porous species differ from those in diffuse-porous species. Species having semi ring porous xylem express high dominance on disturbed areas. Xylem initiation is influenced by buds and leaves, and the timing of xylem initiation and development is different for ring porous and diffuse-porous species. Tress with different anatomical types expresses different levels of sensitivity. Exact mechanisms are yet to be elucidated [44,45]. Studies on the toxicity of nanoparticles in edible plants revealed that not all plants treated with nanoparticles manifested toxicity effects, in fact more studies revealed positive or no consequential effects in plants [46]. There is evidence that MWNTs could translocate from roots to leaves, and fruits and engage in a strong interaction with the cells of tomato seedlings, resulting in significant changes in total gene expression in roots, leaves, and fruits [42]. Conversely, translocation of MWNTs exerts toxic effects of some plants [15,26,47]. Still, the factors associated with the varied toxicological responses of different plant species to nanoparticles have not, yet, been well explored [46]. Canas *et al.* [14] described in their studies that the species would response differently to the nanomaterials, even under the identical experimental conditions. This differential toxicity tentatively suggests that agricultural use of MWNTs may not negatively affect all crop species; positive effects of MWNTs have also been reported [42].

The article "Potential Impact of Multi-Walled Carbon Nanotubes Exposure to the Seedling Stage of Selected Plant Species" was retracted in 2015. Reasons: plagiarized text; duplicated text; overlap with other authors' work; overlap with earlier publications.

Apoptosis and necrosis are two different processes culminating with the in cessation of biological activity. Apoptosis or PCD (programmed cell death) has been defined as a sequence of events that lead to the controlled and organized destruction of the cell. Necrosis, on the other hand, has been described as an uncontrolled form of cell death, which often follows overwhelming cellular stress where the cell is unable to activate its apoptotic pathways [48]. A number of plant adaptation processes, including the HR to pathogens in response to oxygen deprivation, require PCD. In contrast, many unfavorable abiotic stress factors trigger unwanted PCD. Consequently, PCD both serves as a positive and negative aspect of plant adaptation to the environment [49]. One of the earliest events in the HR is a burst of oxidative metabolism leading to the generation of O_2_^−^ and the subsequent accumulation of H_2_O_2_ which has many characteristics in common with PCD or apoptosis [50]. ROS are generated in plants as a result of O_2_ reduction during a number of normal metabolic processes. These harmful and highly reactive intermediates of O_2_ reduction have been considered by many as undesirable by-products of metabolism, and can damage biological molecules and structures [51,52]. Plants initially developed an antioxidant system, consisting of enzymes and nonenzymatic antioxidants as a means of protection against excessive ROS production and adjust ROS levels need at a particular time [53]. The development of this antioxidant system of ROS-producing and -detoxifying enzymes allowed ROS to be co-opted as signaling molecules that regulate various cellular processes, including growth, development, stress adaptation, and cell death. To control so many and such different processes, the biological response to altered ROS levels needs to be very specific. Balancing ROS levels is essential to ensure an accurate execution of their signaling functions and to prevent their toxicity [49]. The fate of the ROS signaling is to a large range related to the chemical properties of different ROS and their doses [49,51]. In general, low doses of ROS protect against oxidative and abiotic stress, while high doses trigger cell death [51]. The oxidative burst is biphasic where the first phase is shorter, having signaling functions, and the second phase is longer with continued ROS production that initiates PCD [50], although extremely high doses of ROS can cause necrosis [54,55]. Therefore, the difference between apoptosis and necrosis may be simply one of timing and severity of insult. Our study shows some of the typical hallmarks of necrosis such as, cell death, loss of membrane integrity and membrane damage.

## 3. Experimental Section

### 3.1. Nanomaterials, Chemicals, and Seeds

MWNTs were purchased (Bayer MaterialScience, Leverkusen, Germany) as powders with a loose agglomerate size of 0.1–1 mm, outer mean diameter ~13 nm, inner mean diameter ~4 nm, and length >1 µm. The powders were first wet with deionized water overnight at ~40 °C, then milled into smaller sizes with a continuously operating bead-mill system in the absence of dispersants (surfactants). The water-wetted milled MWNTs were used throughout this study.

The article "Potential Impact of Multi-Walled Carbon Nanotubes Exposure to the Seedling Stage of Selected Plant Species" was retracted in 2015. Reasons: plagiarized text; duplicated text; overlap with other authors' work; overlap with earlier publications.

Chemicals were purchased from Kanto Chemical Co. Inc. (Hokkaido, Japan), Wako Pure Chemical Industries Ltd. (Tokyo, Japan) and Sigma Aldrich Inc. (Tokyo, Japan). Seeds of lettuce (*Lactuca sativa*), rice (*Oryza sativa* L.), and cucumber (*Cucumis sativus*) were purchased from Sapporo, Japan. Red spinach (*Amaranthus tricolor* L.), lady’s finger (*Abelmoschus esculentus*), and chili (*Capsicum annuum* L.) seeds were purchased from Dhaka, Bangladesh. Professor Toru Miura kindly provided soybean (*Glycine max*) seeds.

### 3.2. Atomic Force Microscopy (AFM), Scanning Electron Microscope (SEM) and Transmission Electron Microscope (TEM)

For AFM, an Agilent Series 5500 AFM instrument (Agilent Technologies, Tokyo, Japan) was used. The samples were prepared by casting a diluted aqueous MWNTs suspension on the surfaces of mica. The images were obtained using the tapping mode at a scanning rate of 1 Hz. For SEM, a few drops of the MWNTs suspension were deposited on the aluminum stub, dried, sputter-coated, and observed using a Hitachi S-4000 SEM (Hitachi, Ibaraki, Japan) with an acceleration voltage of 10 kV. For roots and leaves SEM, the roots and leaves were fixed in 2.5% glutaraldehyde (GA) and 2% paraformaldehyde (PA) in 0.1 M phosphate buffer (PB) buffer (pH 7.4), dehydrated, critical-point dried, sputter-coated, and observed with a Hitachi S-4000 SEM (Hitachi, Ibaraki, Japan). The acceleration voltage was 10 kV. For TEM, a few drops of the suspension were deposited on the TEM grid covered with a Formvar membrane, dried, and evacuated before analysis. The preparations were observed using a Hitachi H-800 TEM. The acceleration voltage was 75 kV.

### 3.3. Hydroponic Culture and Effects of MWNTs on the Growth of the Plants

There is much less evidence on the behavior and toxicity of nanoparticles in terrestrial systems, due to complications in measuring dose and/or dispersion of nanoparticles in the test solutions. In aquatic toxicity testing, the pollutant is usually in true solution and homogeneously distributed throughout the sample. Rico *et al.* [46] pointed out that the knowledge on plant toxicity of nanomaterials is at the foundation stage. Knowledge about their potential toxicity is important before these nanomaterials can be used in actual soil settings. Furthermore, the primary interactions of these nanomaterials with physiological parts of plant is a key feature of understanding their biological impact, and these interactions can perhaps be exploited to mitigate undesirable toxic effects. To conduct toxicity studies in soil media are needed since nanoparticles are likely to react with the constituents of environmental matrices that will enhance, lessen or modify the toxic effect of nanoparticles [46]. Seeds were sterilized, soaked overnight, and incubated at 25 °C, and the seedlings were transferred to plastic pots containing 300 mL Modified Hoagland Media [56] with 0, 20, 200, 1000, or 2000 mg/L MWNTs, with three replicates per treatment. The major factor affecting toxicity in food crops is the concentration of nanoparticle. Rico *et al.* [46] have concluded that nanoparticles showing a manifest toxic effect on the food crops usually appear in the range of concentration of 1000–4000 mg/L. According to USEPA guidelines [57], the highest concentration of MWNTs used for this study was 2000 mg/L. Toxicity studies on the food crops were commonly carried out at high concentrations (2000–5000 mg/L) of the nanoparticles [21,58]. At 1000 and 2000 mg/L, the MWNTs solution was stable with very little settling. Solutions were manually agitated before use. The pH of media was adjusted to 6.0 and remained unchanged with time. After 15 days of hydroponic culture, seedling roots and shoots were separated; the fresh weights were measured and the lengths of individual seedlings were determined.

The article "Potential Impact of Multi-Walled Carbon Nanotubes Exposure to the Seedling Stage of Selected Plant Species" was retracted in 2015. Reasons: plagiarized text; duplicated text; overlap with other authors' work; overlap with earlier publications.

### 3.4. Effect of MWNTs on Cell Death (Evans Blue and Electrolyte Leakage)

The cell death of MWNTs-treated and untreated (control) plant roots was tested as previously described by Baker and Mock [59], using Evans blue after 15 days of MWNT exposure. Root samples were incubated with Evans blue (0.025% *v*/*v*) for 2 h at room temperature (25 °C) and washed with water several times. Cell death was measured spectroscopically after extraction of the Evans blue using 1% (*w*/*v*) SDS (sodium dodecyl sulfate) in 50% (*v*/*v*) methanol at 50 °C for 15 min. The absorbance of the extracted solution was read at a wavelength of 597 nm (V-530 UV/UISNIR Spectrophotometer, Jasco, Tokyo, Japan). Cell death was expressed as absorbance of treated roots in relation to untreated roots (control).

Cell death was evaluated by also measurement of ion leakage from leaves. The percent of membrane injury was measured from the electrolyte leakage of treated and untreated plants by a conductivity method based on the method of Lutts *et al.* [60] with some changes. Leaf samples (100 mg) were taken in test tubes containing 10 mL of distilled water, after three washes with distilled water to remove surface contamination. Test tubes were covered and incubated at room temperature (25 °C) on a shaker (100 rpm) for 24 h. Electrical conductivity of the solution (*L*_t_) was determined. Samples were then autoclaved at 120 °C for 20 min, and a final conductivity reading (*L*_0_) was obtained upon equilibration at 25 °C. Electrolyte leakage was defined as: Electrolyte leakage (%) = (*L*_t_/*L*_0_) × 100. The extent of membrane injury (leakage of electrolytes) from cells was determined with a portable conductivity meter (pH/Cond Meter, Horiba D-54, Horiba, Kyoto, Japan).

The article "Potential Impact of Multi-Walled Carbon Nanotubes Exposure to the Seedling Stage of Selected Plant Species" was retracted in 2015. Reasons: plagiarized text; duplicated text; overlap with other authors' work; overlap with earlier publications.

### 3.5. Detection of ROS (Hydrogen Peroxide, Hydroperoxides, and Superoxide)

We used 3,3'-diaminobenzidine (DAB), to reveal hydrogen peroxide production [61] and we used the fluorogenic probe, 2',7'-dichlorodihydrofluorescin diacetate (DCFH-DA), to detect hydroperoxides inside the cells [62]. We used nitro blue tetrazolium (NBT) salt, a chromogenic redox indicator, to demonstrate the generation and release of superoxide anion [63].

MWNTs-treated (1000 mg/L) and untreated fresh leaves from 15-day-old plants were placed in NBT and DAB-HCl, were incubated under vacuum for 2 h and ~8 h, respectively. An insoluble blue formazon compound was produced when NBT reacted with super oxide, and a deep reddish-brown polymerization product was produced when DAB reacted with H_2_O_2_; both could be visualized under a Transmit Light Microscope BX51 with an Olympus DP72 Camera (Olympus corporation, Tokyo, Japan) after chlorophyll was removed from the leaves by boiling 15 min in ethanol.

DCFH-DA was used for visualization of intracellular ROS by spectroscopy. Fresh leaves were incubated in DCFH-DA for 2 h for detection of ROS. After three PBS (phosphate-buffered saline) rinses, images were captured using fluorescence microscopy (Olympus IX70, Olympus, Tokyo, Japan).

### 3.6. Statistical Analysis

Phytotoxicity endpoints for all measurements were compared to those of the untreated control/unexposed (without MWNTs, only Modified Hoagland Media). Statistical analysis was performed using Student’s *t*-test, with *P* ° 0.01 considered significant. Data are presented as mean ±SD (standard deviation).

## 4. Conclusions

This investigation underscores the importance of effective screening strategies for exposure of agricultural and environmental systems in which MWNTs can penetrate the root and be transported to leaf and fruits [64]. Little is currently known about plant uptake of carbon nanotubes, or about how toxicity is affected by plant type. In the future, long-term studies are necessary to identify target plants and to understand MWNTs-induced phytotoxicity; such studies will be relevant to use and disposal of engineered nanoparticles.
